This article has been retracted.

# LncRNA Gm43843 Promotes Cardiac Hypertrophy via miR-153-3p/Cacna1c Axis

**DOI:** 10.1155/2022/2160804

**Published:** 2022-10-10

**Authors:** Yuhua Cai, Yunpeng Li

**Affiliations:** ^1^Department of Cardiology, Jingzhou First Municipal Hospital, Jingzhou 434000, Hubei Province, China; ^2^Department of Cardiovasology, Dongfeng Hospital, Hubei University of Medicine, Shiyan 442000, Hubei Province, China

## Abstract

Long noncoding RNAs (lncRNAs) have been reported to engage in many human diseases, including cardiac hypertrophy. Cardiac hypertrophy was mainly caused by excessive pressure load, which can eventually lead to a decline in myocardial contractility. Gm43843, a novel lncRNA, has not been well explored in cardiac hypertrophy so far. Herein, we are going to search the function and the underlying molecular mechanism of Gm43843 in cardiac hypertrophy. Gm43843 levels were measured via qRT-PCR in mouse myocardial cells when they are treated with angiogenin II (Ang II) or transfected with different plasmids. Western blot assay was implemented to detect the cardiac hypertrophy-related protein markers, while the cell was analyzed via immunofluorescence (IF) assay to evaluate the hypertrophy. Meanwhile, the binding of Gm43843 and the putative targets was examined based on mechanistic assay results. We found that Gm43843 expression was increased with the elevated concentration of Ang II. Inhibited Gm43843 was detected to reduce the hypertrophy of mouse myocardial cells. Meanwhile, Gm43843/miR-153-3p/Cacna1c axis was found to modulate cardiac hypertrophy. In short, Gm43843 promotes cardiac hypertrophy via miR-153-3p/Cacna1c axis.

## 1. Introduction

Cardiac hypertrophy is a slow but effective compensatory function, which happened under long-term pressure overload [1]. Pathological cardiac hypertrophy poses a high risk of myocardial ischemia, which will lead to a deficiency in myocardial contractility, and eventually causes heart failure [2]. The major treatment for cardiac hypertrophy is surgical therapy [3]. Nevertheless, a lack of knowledge in the pathogenesis of cardiac hypertrophy makes the prevention of this disease difficult [4]. Thence, it has become vitally important for us to explore the underlying molecular mechanism in cardiac hypertrophy.

Noncoding RNAs (ncRNAs) are a group of genes, lacking protein-coding ability, but play important roles in modulating the biological behavior of cells [5–8]. Meanwhile, increasing long ncRNAs (lncRNAs) have been found to have a connection with the progression of cardiac hypertrophy by acting as competing endogenous RNAs (ceRNAs), that is, to sponge microRNAs (miRNAs) and modulate downstream messenger RNA (mRNA) expression [9]. For instance, lncRNA MIAT has been revealed to sequester miR-93 and regulate the expression of TLR4 in cardiac hypertrophy, functionally promoting the progression of cardiac hypertrophy [10]. Additionally, lncRNA MIAT contributes to cardiac hypertrophy by modulating the miR-93/Akt3 axis [11]. LncRNA-ROR can also modulate the progression of cardiac hypertrophy via miR-133 [12]. Gm43843 is a novel lncRNA that has not been well investigated so far. Limited evidence has suggested that lncRNA Gm15834 is allowed to facilitate myocardial hypertrophy by serving as a miR-30b-3p sponge and elevating ULK1 expression [13]. In our study, we are going to search for the function of Gm43843 in cardiac hypertrophy.

MiR-153-3p is a crucial regulator identified in various diseases. Specifically, in cardiac diseases, it has been found that miR-153-3p contributes to mitochondrial fragmentation in cardiac hypertrophy [9]. The regulatory influence of miR-153-3p on cardiomyocyte apoptosis by directly targeting *β*II spectrin has also been uncovered [14]. Recent evidence has also pointed out that miR-153-3p is able to affect cardiomyocyte apoptosis induced by formaldehyde [14]. Herein, we aim to figure out whether miR-153-3p is a participant of the Gm15834-centered ceRNA regulatory axis.

mRNA calcium voltage-gated channel subunit alpha1C (Cacna1c) has been recognized as the effector of a wide range of neuropsychiatric syndromes [15]. Importantly, it has once been revealed that Cacna1c targeted by miR-221/222 is related to the change in cardiac ion channel expression and current density [16]. Cacna1c is also essential for cardiac electrophysiological development and maturation [17]. Therefore, it is one of the major targets of our study to uncover the function of Cacna1c in cardiac hypertrophy. Atrial natriuretic factor (ANF), brain natriuretic peptide (BNP), and *β*-myosin heavy chain (*β*-MHC) have been known as the biomarker of cardiac hypertrophy progression [11, 18]. In our study, these markers were detected to reflect hypertrophy. Meanwhile, the surface area of mouse myocardial cells was also assessed for investigating the hypertrophy variation.

In this study, the specific molecular mechanism of lncRNA Gm43843 in cardiac hypertrophy will be scrutinized, with the ceRNA network taken into consideration.

## 2. Materials and Methods

### 2.1. Cell Culture and Treatment

The mouse myocardial cells (H9C2 and MCM) were available from the ATCC (Manassas, VA). The cell culture environment was kept with 5% CO_2_ at 37°C. Dulbecco's modified Eagle's medium (DMEM) supplemented with 1% antibiotics and 10% fetal bovine serum (FBS) was procured from Gibco (Grand Island, NY). To induce cardiac hypertrophy, H9C2 and MCM cells were severally processed with angiotensin II (Ang II; Sigma–Aldrich, St. Louis, MI) at 0.5 or 1 mmol/L concentration for 48 h.

### 2.2. RNA Extraction and Quantitative Real-Time PCR (qRT-PCR)

Total RNA was isolated from cardiomyocytes utilizing TRIzol reagent (Thermo Fisher Scientific, Waltham, MA), followed by reverse transcription with the application of a reverse transcription system (Thermo Fisher Scientific). qRT-PCR was conducted on ABI 7900 Detection System (Applied Biosystems, Foster City, CA) by use of the SYBR-Green PCR Master Mix kit (Takara, Shiga, Japan). Relative expression of genes, normalized to GAPDH or U6, was calculated via the 2^−ΔΔCt^ approach.

### 2.3. Plasmid Transfection

The synthesized short hairpin RNAs (shRNAs) and control-shRNAs (GenePharma, Shanghai, China) were available to silence Gm43843 and Cacna1c using Lipofectamine3000 (Thermo Fisher Scientific). In addition, the miR-153-3p mimics and NC mimics, miR-153-3p inhibitor and NC inhibitor, as well as the pcDNA3.1-Cacna1c and pcDNA3.1-NC were all available from GenePharma for 48 h of plasmid transfection.

### 2.4. Western Blot

Total protein was extracted from cells by use of RIPA lysis buffer (Beyotime, Shanghai, China). Thereafter, the separation of proteins was achieved by using 10% SDS-PAGE (Bio-Rad, Hercules, CA), and the samples were then moved to PVDF membranes (Millipore, Bedford, MA). Following sealing with 5% fat-free milk, the membranes were cultivated at 4°C overnight with primary antibodies for ANP (1 : 2000; Abcam, Cambridge, MA), BNP (1 : 2000; Abcam), *β*-MHC (1 : 2000; Abcam) and control GAPDH (1 : 2000; Abcam). Later, secondary antibodies (1 : 5000; Abcam) were added to the culture for 1 h at 37°C. Finally, proteins were evaluated by the ECL detection system (Pierce, Rockford, IL, USA).

### 2.5. Immunofluorescence (IF)

Processed H9C2 and MCM cells were fixed utilizing cold methanol (Sigma–Aldrich), followed by incubation with primary antibodies against *α*-actin (Abcam) and secondary antibodies conjugated to Alexa Fluor 488. Images were at last taken via fluorescence microscope (Olympus, Tokyo, Japan). After randomly examining 50 cells in 3 independent experiments, we obtained the average value for analyses. Image-Pro Plus 6.0 software was used to evaluate the surface area.

### 2.6. Fluorescence In Situ Hybridization (FISH)

The subcellular localization of Gm43843 was examined through the FISH kit (Roche, Mannheim, Germany). Cells were cultured with a hybridization solution containing a specific Gm43843 probe (Sigma–Aldrich). The nuclei were dyed in DAPI (Sigma–Aldrich) for 10 min. At last, cells were captured via a fluorescence microscope to record images of fluorescence.

### 2.7. Subcellular Fraction

Nuclear/cytoplasmic fractionation PARIS Kit (Thermo Fisher Scientific) was used for collecting nuclear and cytoplasmic fractions of cells. The qRT-PCR was performed to determine the relative expression of Gm43843, GAPDH (cytoplasmic reference), and U6 (nuclear reference).

### 2.8. Luciferase Reporter Assay

The wild-type and mutated Gm43843 or Cacna1c fragments covering miR-153-3p binding sites were subcloned into pmirGLO dual-luciferase vector (Promega, Madison, WI). The acquired Gm43843-WT/Mut and Cacna1c-WT/Mut reporter vectors were cotransfected into cells with miR-153-3p mimics or NC mimics for 48 h. Luciferase activity was measured with a dual-luciferase reporter assay system (Promega).

### 2.9. RNA Pull Down

The wild-type and mutated miR-153-3p fragment covering Gm43843 or Cacna1c binding sites were labeled separately with biotin into Bio-miR-153-3p-WT/Mut probes. Biotinylated RNA was incubated with cell lysates and magnetic beads, and the RNAs in the complexes pulled down were purified and detected by qRT-PCR.

### 2.10. Bioinformatics Prediction

StarBase website (https://starbase.sysu.edu.cn/) was employed for projecting candidate miRNAs targeted by Gm43843 with no specific condition. This database was also applied for screening potential mRNA likely binding with miR-153-3p in the subset of microT. The potential binding sequences of Gm43843 and Cacna1c covering miR-153-3p binding sites were obtained from starBase as well.

### 2.11. Statistical Analysis

All assays were run thrice. Values were shown as mean ± SD. GraphPad Prism 7 software (GraphPad Software, La Jolla, CA, USA) was utilized for statistical analysis with Student's *t*-test for two groups or one-way/two-way ANOVA for three or more groups with one or two variables. Tukey and Dunnett's approaches were applied as post hoc tests. The level of significance was specified as *p* < 0.05.

## 3. Results

### 3.1. Inhibited Gm43843 Relieved Cardiac Hypertrophy

Reportedly, lncRNAs play vital parts in the progression of cardiac hypertrophy [10, 19, 20]. Herein, we discussed the role of lncRNA Gm43843 in cardiac hypertrophy. Above all, it was noticed that Gm43843 expression increased upon the elevation of Ang II concentration in mouse myocardial cells (H9C2 and MCM) (Figure 1(a)). Thence, we predicted that Gm43843 played its regulatory function in H9C2 and MCM cells. Furthermore, inhibition efficiency of Gm43843 was detected via qRT-PCR assay (Figure 1(b)). As presented in Figures 1(c)-1(d), Ang II (1 mmol/L) significantly increased the mRNA and protein levels of the biomarkers of cardiac hypertrophy (ANF, BNP, and *β*-MHC) in H9C2 and MCM cells. When Gm43843 was inhibited, their expressions were decreased. These findings indicated that Ang II (1 mmol/L) induced H9C2 and MCM cell hypertrophy. However, Gm43843 inhibition decreased the hypertrophy symptom. Meanwhile, the IF assay assessed the cell surface area (Figure 1(e)). Results found that cell surface area expanded after Ang II (1 mmol/L) treatment, but reduced again by silenced Gm43843. In conclusion, inhibited Gm43843 relieved cardiac hypertrophy.

### 3.2. MiR-153-3p Could Bind to Gm43843 in H9C2 and MCM Cells

It has been scrutinized that cytoplasmic lncRNAs can function as ceRNAs to regulate downstream RNA expression [21]. In our study, we firstly investigated the location of Gm43843 in H9C2 and MCM cells (Figures 2(a)-2(b)). We could see from the result that Gm43843 was mainly located in the cytoplasm in H9C2 and MCM cells. Thence, we further searched the miRNAs that were predicted to bind to Gm43843 via the starBase website and their expressions were assessed in H9C2 and MCM cells treated with Ang II (1 mmol/L) (Figure 2(c)). We could see that mmu-miR-153-3p was down-regulated in H9C2 and MCM cells upon Ang II (1 mmol/L) treatment. Meanwhile, the binding site of Gm43843 and mmu-miR-153-3p was manifested based on starBase prediction (Figure 2(d)). After the high miR-153-3p overexpression efficiency was verified (Figure 2(e)), we confirmed the binding relationship between Gm43843 and miR-153-3p as the luciferase activity of Gm43843-WT was weakened due to miR-153-3p augmentation (Figure 2(f)). RNA pull-down assay further supported the above finding, since Bio-miR-153-3p-WT probes largely pulled down Gm43843 but Bio-miR-153-3p could not (Figure 2(g)). To sum up, miR-153-3p is directly targeted by Gm43843 in H9C2 and MCM cells.

### 3.3. Cacna1c Is Able to Combine with miR-153-3p in H9C2 and MCM Cells

In this part, we further explored the target gene of miR-153-3p to complete the ceRNA network. According to the starBase website, we found 700 mRNAs in the subset of microT. All of these mRNAs were implemented into qRT-PCR assay to detect the most suitable mRNA whose expression could be affected by inhibited Gm43843 and overexpressed miR-153-3p in H9C2 cells with or without Ang II treatment (Figure 3(a)). Xkr4 and Cacna1c were found. Meanwhile, the expression of Xkr4 and Cacna1c was investigated with different concentrations (0.5 and 1 mmol/L) of Ang II in H9C2 and MCM cells via qRT-PCR assay (Figure 3(b)). We detected that only Cacna1c expression increased with the elevation of Ang II concentration. Thence, Cacna1c was selected as the target. We presented the binding site of Cacna1c and mmu-miR-153-3p (Figure 3(c)). The binding affinity between Cacna1c and mmu-miR-153-3p was corroborated, as the wild type of Cacna1c luciferase activity was observed to be reduced on account of miR-153-3p up-regulation (Figure 3(d)). Cacna1c was also substantially pulled down by the wild type of Bio-miR-153-3p in H9C2 and MCM cells (Figure 3(e)). In a word, Cacna1c could bind to miR-153-3p in H9C2 and MCM cells.

### 3.4. Cacna1c Inhibition Could Relieve the Hypertrophy of H9C2 and MCM Cells

Previous studies have claimed the function of Cacna1c in the progression of cardiomyocyte hypertrophy [22–24]. In our study, we further investigated the function of Cacna1c in H9C2 and MCM cells. We first knocked down Cacna1c in H9C2 and MCM cells (Figure 4(a)). Then, we found that ANF, BNP, and *β*-MHC expressions were both inhibited by silenced Cacna1c (Figures 4(b)-4(c)). Meanwhile, the IF assay delineated that cell surface area was reduced when Cacna1c was inhibited in H9C2 and MCM cells (Figure 4(d)). To conclude, Cacna1c inhibition could relieve the hypertrophy of H9C2 and MCM cells.

### 3.5. Gm43843/miR-153-3p/Cacna1c Axis Could Modulate the Hypertrophy of H9C2 and MCM Cells

We further studied the function of the Gm43843/miR-153-3p/Cacna1c axis in cardiac hypertrophy. We found that Cacna1c expression was significantly decreased with the silencing of Gm43843, but recovered with the inhibition of miR-153-3p (Figure 5(a)). After that, we overexpressed Cacna1c and the overexpression efficiency was proved to be high (Figure 5(b)). It was detected that RNA expressions and protein levels of ANF, BNP, and *β*-MHC were inhibited by Gm43843 depletion, but then, they were rescued by miR-153-3p inhibition or Cacna1c overexpression (Figures 5(c)-5(d)). Meanwhile, the IF assay found that lessened cell surface area due to knockdown of Gm43843 was increased again after miR-153-3p inhibition or Cacna1c augment (Figure 5(e)). In conclusion, Gm43843 could modulate the hypertrophy of H9C2 and MCM cells through miR-153-3p/Cacna1c.

## 4. Discussion

Accumulating evidence has proved that lncRNA can play regulating roles in cardiac hypertrophy. For example, Plscr4 increment can reduce Ang II-induced cardiomyocyte hypertrophy by regulating the expression of miR-214 and Mfn2 [25]. LncRNA CASC15 upregulated in cardiomyocytes treated with Ang II can increase the cell surface area of cardiomyocytes in cardiac hypertrophy by modulating the miR-432-5p/TLR4 pathway [26]. Meanwhile, H19 inhibition can activate cardiomyocyte hypertrophy, and H19 can regulate miR-675 targeting CaMKII*δ* in cardiac hypertrophy [27]. In our study, we searched the role of Gm43843 in mouse myocardial cells treated with Ang II for inducing hypertrophy. Gm43843 expression was found up-regulated with the Ang II concentration increasing. Furthermore, Gm43843 inhibition was observed to relieve the cardiac hypertrophy of mouse myocardial cells. Meanwhile, the IF assay reassured that silenced Gm43843 played an inhibitory role in cardiac hypertrophy.

Previous studies have reported the ceRNA character of lncRNAs, which indicated that lncRNAs can function as miRNA sponges to form a miRNA/mRNA pathway to modulate the progression of human disease [28–30]. For example, lncRNA HOXD-AS1 can sponge to miR-130a-3p activating the expression of SOX4 to enhance the progression of liver cancer [31]. LncRNA TDRG1 can modulate cervical cancer cell growth, migration, and invasion via the miR-326/MAPK1 axis [32]. In our study, we firstly located Gm43843 in the cytoplasm in mouse myocardial cells. Mmu-miR-153-3p was corroborated to bind to Gm43843. Furthermore, Cacna1c was validated to bind to mmu-miR-153-3p.

Increasing molecular genetic testing has suggested that Cacna1c-linked disorders account for pathogenic variants and clinical findings. Cacna1c is related to calcium channel function and individuals with a pathogenic variant of this gene have a risk for cardiovascular disease [33]. Specifically, previous studies have unveiled that Cacna1c was involved in the progression of cardiomyocyte hypertrophy [22–24]. CACNA1C expression could be inhibited by miR-135b in cardiomyocytes to relieve the symptom of pathological cardiac hypertrophy [23]. In our study, we found the expression of Cacna1c was up-regulated with Ang II inducement. It was worth noting that Cacna1c inhibition decreased the expression and protein level of ANF, BNP, and *β*-MHC, as well as reduced the cell surface area of mouse cardiomyocytes. Last but not least, it was verified that miR-153-3p inhibition or Cacna1c augmentation was able to abrogate the suppressive impact of Gm43843 deficiency on the hypertrophy of mouse cardiomyocytes.

To conclude, Gm43843 promotes cardiac hypertrophy via miR-153-3p/Cacna1c axis. Although human cells and clinical samples need to be involved in the future study for further confirmation of the validity of the axis, our study can still provide a novel perspective for a more in-depth understanding of the molecular mechanism in cardiac hypertrophy.

## Figures and Tables

**Figure 1:** Inhibited Gm43843 relieved cardiac hypertrophy. (a) Gm43843 expression was detected via qRT-PCR assay when mouse myocardial cells (H9C2 and MCM) were treated with Ang II. (b) The inhibition efficiency of Gm43843 was monitored via qRT-PCR assay in H9C2 and MCM cells with or without the treatment of Ang II. (c-d) QRT-PCR assay and western blot assay were implemented to detect ANF, BNP, and *β*-MHC expression at mRNA and protein levels. (e) IF assay examined the variation of H9C2 and MCM cell surface. ^*∗∗*^*P* < 0.01.

**Figure 2:** Gm43843 sequesters miR-153-3p in H9C2 and MCM cells. (a-b) The location of Gm43843 was investigated by FISH assay and subcellular fraction assay in H9C2 and MCM cells with or without Ang II treatment. (c) Thirteen miRNA candidates were searched from the starBase website, and their expression was detected in H9C2 and MCM cells treated with Ang II (1 mmol/L) via qRT-PCR assay. (d) The wide-type and mutated binding sites of Gm43843 and mmu-miR-153-3p were presented based on starBase prediction. (e) The overexpression efficiency of miR-153-3p was verified by qRT-PCR assay. (f-g) Luciferase reporter assay and RNA pull-down assay evaluated the binding relationship between Gm43843 and mmu-miR-153-3p. ^*∗∗*^*P* < 0.01.

**Figure 3:** Cacna1c could bind to miR-153-3p in H9C2 and MCM cells. (a) QRT-PCR assay examined the most suitable mRNA whose expression could be affected by inhibited Gm43843 and overexpressed miR-153-3p in H9C2 cells. (b) Xkr4 and Cacna1c mRNA levels were investigated in H9C2 and MCM cells via qRT-PCR assay with the treatment of different concentrations (0.5 and 1 mmol/L) of Ang II. (c) The binding site of Cacna1c and mmu-miR-153-3p was displayed on the basis of starBase prediction. (d-e) Luciferase reporter and RNA pull-down assays reassured the binding in Cacna1c and mmu-miR-153-3p. ^*∗*^*P* < 0.05, ^*∗∗*^*P* < 0.01.

**Figure 4:** Cacna1c inhibition relieves the hypertrophy of H9C2 and MCM cells. (a) The inhibition efficiency of sh-Cacna1c was investigated by qRT-PCR assay in cells treated with Ang II. (b-c) QRT-PCR assay and western blot assay were implemented to detect the hypertrophy-related protein markers in Ang II-treated H9C2 and MCM cells upon Cacna1c depletion. (d) IF assay revealed the changes in H9C2 and MCM cell surface when Cacna1c was inhibited. ^*∗∗*^*P* < 0.01.

**Figure 5:** Gm43843/miR-153-3p/Cacna1c modulates the hypertrophy of H9C2 and MCM cells. (a) Cacna1c level variation upon Gm43843 depletion and miR-153-3p inhibition in Ang II-treated cells was evaluated via qRT-PCR. (b) Overexpression efficiency of Cacna1c was detected by qRT-PCR assay in cells after Ang II treatment. (c-d) The expression of ANF, BNP, and *β*-MHC at mRNA or protein levels was analyzed. (e) IF assay detected the surface of H9C2 and MCM cells. ^*∗∗*^*P* < 0.01.

## Data Availability

The data used in this study are presented in the manuscript.
